# RC-3095, a Selective Gastrin-Releasing Peptide Receptor Antagonist, Does Not Protect the Lungs in an Experimental Model of Lung Ischemia-Reperfusion Injury

**DOI:** 10.1155/2015/496378

**Published:** 2015-03-29

**Authors:** Vera L. Oliveira-Freitas, Leonardo Dalla Giacomassa Rocha Thomaz, Lucas Elias Lise Simoneti, Christiane Malfitano, Kátia De Angelis, Jane Maria Ulbrich, Gilberto Schwartsmann, Cristiano Feijó Andrade

**Affiliations:** ^1^Department of Research Group and Post-Graduation, Hospital de Clínicas de Porto Alegre, Ramiro Barcelos 2350, Sala 2227, 90.035-903 Porto Alegre, RS, Brazil; ^2^Lung and Airway Laboratory, Federal University of Rio Grande do Sul, Hospital de Clínicas de Porto Alegre, Ramiro Barcelos 2350, Sala 21313, 90.035-903 Porto Alegre, RS, Brazil; ^3^Laboratory of Translational Physiology, Universidade Nove de Julho, Rua Vergueiro 235/249, 3 Subsolo, 01.504-000 São Paulo, SP, Brazil; ^4^Department of Pathology, Hospital de Clínicas de Porto Alegre, Ramiro Barcelos 2350, 90.035-903 Porto Alegre, RS, Brazil; ^5^Department of Internal Medicine, Faculty of Medicine, Federal University of Rio Grande do Sul, Hospital de Clínicas de Porto Alegre, Rua Ramiro Barcelos 2350, 3° Leste, 90.035-903 Porto Alegre, RS, Brazil; ^6^Department of Thoracic Surgery, Hospital de Clínicas de Porto Alegre and Hospital da Criança Santo Antônio, Ramiro Barcelos 2.350, 90035-903 Porto Alegre, RS, Brazil

## Abstract

RC-3095, a selective GRPR antagonist, has been shown to have anti-inflammatory properties in different models of inflammation. However, its protective effect on lungs submitted to lung ischemia-reperfusion injury has not been addressed before. Then, we administrated RC-3095 intravenously before and after lung reperfusion using an animal model of lung ischemia-reperfusion injury (LIRI) by clamping the pulmonary hilum. Twenty Wistar rats were subjected to an experimental model in four groups: SHAM, ischemia-reperfusion (IR), RC-Pre, and RC-Post. The final mean arterial pressure significantly decreased in IR and RC-Pre compared to their values before reperfusion (*P* < 0.001). The RC-Post group showed significant decrease of partial pressure of arterial oxygen at the end of the observation when compared to baseline (*P* = 0.005). Caspase-9 activity was significantly higher in the RC-Post as compared to the other groups (*P* < 0.013). No significant differences were observed in eNOS activity among the groups. The groups RC-Pre and RC-Post did not show any significant decrease in IL-1*β* (*P* = 0.159) and TNF-*α* (*P* = 0.260), as compared to IR. The histological score showed no significant differences among the groups. In conclusion, RC-3095 does not demonstrate a protective effect in our LIRI model. Additionally, its use after reperfusion seems to potentiate cell damage, stimulating apoptosis.

## 1. Introduction

Lung ischemia reperfusion injury (LIRI) is the main cause of early graft dysfunction and death after lung transplantation [1]. Pulmonary edema constitutes its most frequent clinical manifestation, which is triggered by an excessive release of proinflammatory mediators, reactive oxygen species (ROS), cytokines, and neutrophil infiltration in the lungs [2–4]. Ischemia causes an imbalance between metabolic supply and demand, leading to tissue hypoxia, cellular damage, and death [5].

Several methods and substances have been used as an attempt to protect the lungs during the early phase of posttransplantation and to improve short- and long-term graft performance; however, these efforts have generated limited results [6, 7]. The techniques include lung protective ventilation [8, 9], appropriate fluid management, the optimization of organ preservation in lung transplantation, and the minimization of ventilation and anoxic ischemic time [10].

The gastrin-releasing peptide (GRP) is a neuropeptide that acts through G protein-coupled receptors [11]. It participates in signal transmission in both the central and peripheral nervous systems [11, 12]. Its preferred receptor, gastrin-releasing peptide receptor (GRPR), is expressed by various cell types, including those of the gastric, respiratory, and nervous systems, and it is overexpressed in tumor cells [12]. Recent studies have demonstrated the relationship between GRPR signaling and inflammation [13]. GRPR is involved in the induction of innate and adaptive immune responses by inducing mast cell chemotaxis, macrophage migration, and T cell and fibroblast proliferation [14].

RC-3095, a selective GRPR antagonist, has been shown to have anti-inflammatory properties in murine models of arthritis, gastritis, uveitis, and sepsis by attenuating the release of proinflammatory cytokines such as tumor necrosis factor-alpha (TNF-*α*) and interleukin-1-beta (IL-1*β*) and the activation and migration of mononuclear cells to sites of inflammation [15]. In addition, GRP mediates air pollution-induced airway hyperreactivity and inflammation in rodents [13].

Because GRPR signaling has been shown to be a relevant component of the inflammatory response in various experimental models and the excessive release of proinflammatory mediators and cytokines, as well as neutrophil infiltration in the lung, is a central event for the development of LIRI, we hypothesized that the GRPR antagonist, RC-3095, imparts a protective effect on LIRI.

## 2. Materials and Methods

The animals were handled in accordance with the Animal Welfare Act and the Guidelines for the Care and Use of Laboratory Animals (NIH Publication, revised 1996). The Ethical Committee of the Hospital de Clínicas de Porto Alegre approved the experimental protocols.

### 2.1. Experimental Protocol

Twenty Wistar male rats with a mean weight of 360 g were randomly assigned to one of four treatment groups (*n* = 5): simulation of surgery (SHAM), ischemia-reperfusion (IR), RC-Pre (RC-3095 Pre-LIRI), and RC-Post (RC Post-LIRI). RC-3095 was administered as a single dose to the left jugular vein 15 min before the induction of ischemia (RC Pre-IR group) and immediately after clamp removal (RC Post-IR group). All animals were observed for 120 min after reperfusion. RC-3095 (0.3 mg/1 mL) was diluted in normal saline, following the protocol described in previous studies conducted by our research group [13].

The animals were subjected to induction anesthesia with 0.5 L/min of oxygen flow and isoflurane (100 mL/min). Rats were systemically heparinized (1 mg/kg) parenterally and underwent cervical tracheostomy with a plastic cannula (Abbocath #14, Abbott Laboratories, Abbott Park, IL, USA).

Anesthesia was then maintained using 0.2 L/min of oxygen flow and isoflurane (10 mL/min). The animals were mechanically ventilated with room air (Harvard Rodent Ventilator, Model 683, Harvard Apparatus Co., Millis, MA, USA) using a tidal volume of 8 mL/kg body weight, a respiratory rate of 70–80 breaths/min, and a positive end-expiratory pressure of 2 cm H_2_O.

The mean arterial pressure (MAP) was measured through cannulation of the right carotid artery (Sirecust 730, Siemens, Solna, Sweden), which was also used for collecting samples for arterial blood gas analysis (Blood Gas Analyzer, Siemens Bayer 865, Siemens).

Left thoracotomy was performed in the fifth intercostal space, the pulmonary ligament was sectioned, and subsequently, the left pulmonary hilum was clamped (Vicca Neuroclip, Cachoeirinha, RS, Brasil). Immediately before clamping, lung expansion was achieved through occlusion of the expiratory valve for three inspiratory cycles to prevent alveolar collapse and consolidation. During the clamping period, both lungs were maintained on mechanical ventilation using the settings previously described [16].

MAP and arterial blood gases were measured before thoracotomy (baseline), after ischemia (predetermined 45-min), and at the end of the experiment. After the 120 min reperfusion period, the animals were sacrificed by incision of the abdominal aorta. Hemodynamic, gas exchange, and pulmonary mechanics were measured at baseline, after lung injury, and after 120 min of observation.

### 2.2. Measurement of Cytokine Levels

Tissues of the right and left lungs were sectioned, weighed, and stored at −80°C. Homogenates were prepared by incubating the tissues in a tissue lysis buffer containing 10% Triton X-100 dissolved in a solution consisting of 100 mM Tris (pH 7.5), 10 mM EDTA, 100 mM sodium fluoride, 100 mM sodium pyrophosphate, 10 mM sodium orthovanadate, 10 *μ*g/mL aprotinin, 1 *μ*g/mL leupeptin, and 2 mM PMSF, for 30 min on ice. Immediately after incubation, the samples were centrifuged at 13,000 rpm, 4°C for 20 min. The supernatants were submitted for protein quantification by the Bradford method [17], using a standard curve from 50 to 1,000 *µ*g/mL of bovine serum albumin and the Bradford reagent (0.01% coomassie brilliant blue, 47% ethanol, 8.5% phosphoric acid, and distilled water q.s.p); the absorbance was determined at a wavelength of 595 nm.

Protein quantification and expression analysis of IL-1*β* and TNF-*α* were performed using an enzyme-linked immunosorbent assay (ELISA) method that was specific for each cytokine. The ELISA protocol was performed with the Duo-set (BD Bioscience Inc., MA, USA).

### 2.3. Immunohistochemical Studies

Caspase-9 and eNOS activity were performed on serial sections prepared from paraffin-embedded, formalin-fixed rat lungs. After paraffin removal using xylene, the sections were rehydrated and subjected to a 40 min to heat treatment at 80°C. The specimens were incubated in a peroxidase block reagent (BIOGEN) to quench endogenous peroxidase activity and any nonspecific reaction was blocked for 10 min.

The sections were then incubated with primary antibodies specific for caspase-9 and eNOS (Asp353, Cell Signaling) and (H-159-Santa Cruz), respectively, at a dilution of 1 : 100, for 2 h at room temperature, followed by incubation with the labeled polymer for 30 min. Staining was performed by incubating the sections with diaminobenzidine tetrahydrochloride substrate chromogen (DAB-BIOGEN), which resulted in a brown-colored precipitate at the antigen site. The sections were then counterstained with hematoxylin for visualization.

Immunohistochemical staining was scored according to the distribution of expression of the target proteins in the evaluated areas, namely, the nucleus, membrane, or cytoplasm. In addition, the intensity of immunostaining was described as follows: 1 = mild, 2 = moderate, and 3 = strong. A semiquantitative approach was used to measure the areas and the intensity of staining of the tissues. A pathologist who was blinded to the clinical and histopathologic information independently analyzed the slides. Caspase-9 and eNOS activity were assed using a cellSens Digital Imaging Software (DP77 microscopy camera, BX41 Microscopy, Olympus).

### 2.4. Histologic Analysis

*Sample Preparation*. The sections of the right and left lungs were excised and then immersed directly in 10% formalin for 60 h; no inflation fixation method was performed. After fixation, the lungs were separated at the hilum, and each lung was sectioned horizontally (right and left lung). The tissue blocks were cut from each region and embedded in paraffin wax, from which 5 mm sections were prepared, mounted, and stained with hematoxylin-eosin.

Two pathologists who were blinded to the experimental protocol, the test groups, and the region of sampling performed the quantitative examination by light microscopy. Each sample was examined under both low and high power fields, and 20 fields from each section were analyzed by one of the pathologists. The other pathologist randomly selected and analyzed those 20 fields from each sample.

The severity of histologic lesions was assed using a score (HIS) that was based on six parameters: intra-alveolar edema, hyaline membrane formation, hemorrhage, recruitment of granulocytes into the air space, focal alveolar collapse or consolidation, and epithelial desquamation/necrosis of airways or alveoli. Each parameter was evaluated semiquantitatively using the following scale: 0 = absent, 1 = mild, 2 = moderate, and 3 = prominent. In addition, the percentage of the involved area of each histologic specimen was estimated (0 to 100%) to quantify any observed histologic changes [18].

For each sample, a weighted histologic score (WIS) was computed from the product of HIS and the percentage of area involved. The HIS and WIS scores of the dependent and nondependent lung regions of each animal were calculated.

### 2.5. Statistical Analysis

The results presented in the text, tables, and figures were expressed as the median ± interquartile range. The data were analyzed using the SPSS version 16.0 statistical software (SPSS Inc., Chicago, IL, USA). Nonparametric Kruskal-Wallis test was performed, followed by chi-squared test for intergroup comparisons. A *P* value of <0.05 was considered significant

## 3. Results

The final mean arterial pressure significantly decreased in the IR and RC Pre-IR groups compared to the baseline (*P* < 0.001). The RC Post-IR group showed a significant decrease in the partial pressure of arterial oxygen at the end of the observation period compared to the baseline (*P* = 0.005) (Table 1).

No differences in the levels of IL-1*β* (*P* = 0.159) and TNF-*α* (*P* = 0.260) were observed in the RC-Pre and RC-Post groups, compared to the IR group (Figure 1).

No significant differences in histological scores were observed among the study groups. The RC-Post group showed a slight reduction in the histological scores compared to that of the other groups (Figure 2).

The caspase-9 activity of pneumocytes was significantly higher in the RC Pos-IR group, compared to the other groups (*P* < 0.013) (Figures 3 and 4). No significant differences in eNOS activity were observed among the groups.

## 4. Discussion

Several studies using both animals and humans have investigated the effects of pharmacologic interventions in reducing the release of proinflammatory cytokines and chemokines, as well as other events that are potentially related to the development LIRI; however, these efforts have generated unclear results [6, 16, 19, 20]

A rodent model for LIRI was selected for the present study because this has been extensively used in the previous reports [16, 21]. This animal model mimics several features of LIRI such as the inflammatory changes and structural damage to the lungs [20, 21]. Furthermore, the differences in mean arterial pressure prior to and after reperfusion among the groups were similar compared to those described in the literature [20].

Only the RC Post-IR group showed a significant decrease in the mean measurements of partial pressure of arterial oxygen at the end of the observation, as compared to the baseline. These results indicate that RC, when administered after reperfusion, potentiates the harmful effects of the IR process.

Although, the present study did not show a clear protective effect of RC on the lung ischemia reperfusion injury model, we observed a trend in reduction of IL-1*β* in the RC-Pre group, compared to that in the IR group. This effect of RC reduction of inflammatory mediators has been demonstrated in various conditions such as arthritis, colitis, and sepsis [22–24]. Unfortunately, information on the level of GRPR expression in the tissues and the GRP levels in plasma was not available for inclusion in the analysis of the present study. This information might have assisted in the interpretation of our results. It is also possible that the basic mechanisms involved in the pathogenesis of LIRI differ from those of other inflammatory conditions whose GPRR signaling could be more relevant [22–24]. Additionally, there are also species-specific pharmacological effects that could sometimes lead to discrepancies between laboratory observations and the findings obtained from patients with LIRI in the clinical setting [1–4, 10].

RC-3095 was administered to animals as a single dose before the induction of ischemia and immediately after clamp removal. This treatment schedule and doses were comparable to those applied by our group in previous studies performed in rodent models [22, 23]. Thus, we could argue that the experimental conditions were adequate for the evaluation of the protective effects of the GRPR antagonist, particularly in terms of dose intensity.

Although GRPR inhibition did not impart a protective effect on our LIRI model, caspase-9 activity in pneumocytes was significantly higher in the animals that received RC-3095 Pos-IR, compared to the other groups. Active caspase-9 cleaves and activates caspase-3, thereby inducing events that lead to DNA fragmentation and cell death. This occurs as early as 15 min after treatment. Thus, once caspase-9 is activated, a protease cascade is initiated, which in turn leads to the rapid activation of caspase-3 and apoptosis [25]. Based on these findings, we hypothesize that, in the presence of RC-3095, caspase-9 was upregulated in the RC-Post group, which activated caspase-3 and resulted in apoptosis as a response mechanism to tissue injury. Interestingly, the RC-Pre group did not show these alterations, suggesting that its administration prior to reperfusion might have a beneficial effect or at least did not induce an increase in caspase-9 activity. Additionally, in a previous study conducted by our group, we observed an increase in the activity of caspase-3 after 45 min of ischemia, which was associated with a higher number of apoptotic cells [21].

eNOS activity mainly observed in the cytoplasm of the endothelial layer of the lung tissue, with a similar distribution among all groups. This finding therefore demonstrates that this enzyme does not have any function in LIRI [26].

In conclusion, the administration of RC3095, which is a selective GRP receptor antagonist, after reperfusion is harmful to IR lungs, as indicated by the induction of apoptosis and the decrease in PaO_2_; however, no signs of lung damage were evident during lung histological analysis. Further studies are necessary to establish the mechanism of GRPR antagonist modulation in the setting of LIRI.

## Figures and Tables

**Figure 1:** IL-1*β* and TNF-*α* protein expression. There was no significant differences in lung tissue protein expression among the groups in IL-1*β* (*P* = 0.159) and TNF-*α* (*P* = 0.260). Data are presented as median ± standard error of the median.

**Figure 2:** Photomicrograph of the lung in the different experimental groups. The histological score (HIS) showed no significant difference between groups (*P* = 0.973) (A: SHAM, B: IR, C: RC-Pre, and D: RC-Post, magnification ×100).

**Figure 3:** Immunohistochemical staining for Cleaved Capase 9. There was maximum expression of brown-positive cells in pneumocytes specially in the RC- POST group (d). ((a): SHAM; (b): IR; (c):RC-PRE; and (d): RC-POST, magnification ×200).

**Figure 4:** Cleaved caspase-9 pneumocyte expression in lung tissues. The RC-Post group exhibited a significant overexpression of cleaved caspase-9 (*P* < 0.013) compared to the other groups. Data are presented as the median ± standard error of the median.

**Table 1:** Hemodynamic variables and gas exchange. Comparative analysis of the groups regarding the time during all experimental protocol.

	MAP			*P*	PaO_2_			*P *	PaCO_2_			*P*
	Baseline	t2	Final		Baseline	t2	Final		Baseline	t2	Final	
SHAM	94 [90; 140]	90 [75; 103]	86 [73.5; 90]	0.165	342.2 [265.2; 353.9]	278.6 [231.4; 300.5]	300.6 [255.95; 378.15]	0.368	47.4 [44.6; 49.9]	44.9 [43.7; 48.9]	47.5 [45.45; 50.8]	0.779

IR	110^*^ [96; 151]	81 [73; 90]	65^**^ [64; 75]	0.007	187.1 [148.6; 318.4]	228.1 [171.9; 348]	149.1 [147.4; 161.2]	0.449	35.9 [32.5; 44.9]	39.9 [34.1; 44.4]	20.7 [20.5; 49.7]	0.819

RC-PRE	93^*^ [85.5; 125]	67.5 [62; 73]	46^**^ [45; 53]	0.015	282.3 [251.2; 341.7]	223.7 [204.4; 394.4]	116.5 [88.7; 269.3]	0.074	41.2 [37.9; 44]	36.7 [34.1; 37]	46.4 [38.4; 50.8]	0.091

RC-POST	86.5 [80.3; 117.3]	76 [72.5; 77]	61.5 [51; 73]	0.105	289.05 [268.5; 294.4]	208.1 [194; 218.9]	181.6 [103.75; 229.5]	0.050	47.5 [40.9; 49.8]	52.3 [50.7; 66.85]	51.25 [49.75; 69.9]	0.174

General	94^∗#^ [85.5; 140]	76^**^ [68; 90]	65^##^ [50; 75]	<0.001	288.2^*^ [199.2; 324.6]	228.1 [199.2; 324.6]	195.3^**^ [129.4; 271.9]	0.005	44.6 [36.6; 49.4]	43.7 [36.7; 43.7]	48.7 [33.9; 51.5]	0.801

The values are described as median ± interquartile range. SHAM group did not have reperfusion and was observed for 120 minutes. t2: five minutes after reperfusion. Final: 120 minutes after reperfusion. The same symbols represent statistically significant difference. MAP = mean arterial pressure; PaO_2_ = partial pressure of arterial oxygen; PaCO_2_ = partial pressure of arterial carbon dioxide. ^∗^ *P* ≤ 0.05.
